The article "Nonlinear Network Speech Recognition Structure in a Deep Learning Algorithm" was published in 2022. Journal: Comput Intell Neurosci.

# Nonlinear Network Speech Recognition Structure in a Deep Learning Algorithm

**DOI:** 10.1155/2022/6785642

**Published:** 2022-03-24

**Authors:** Liang Meng, Prakash Kuppuswamy, Jinal Upadhyay, Sumit Kumar, Shashikant V. Athawale, Mohd Asif Shah

**Affiliations:** ^1^Jilin Agricultural Science and Technology University, Jilin 132101, China; ^2^Department of Computer and Network Engineering, College of Computer Science & Information Technology, Jazan University, Jazan, Saudi Arabia; ^3^Department of Computer Engineering, Alpha College of Engineering and Technology, Gujarat Technological University, Gujarat, India; ^4^Indian Institute of Management, Kozhikode, India; ^5^Department of Computer Engineering, AISSMS COE, Savitribai Phule Pune University, Pune, India; ^6^Kebri Dehar University, Kebri Dehar, Ethiopia

## Abstract

As a result of the fast rise of globalization, people in China are learning English at a rapid pace. However, there is a severe shortage of English teachers in the region, which is a major hindrance. To address these concerns, a deep learning-based algorithm is proposed that can not only check English pronunciation but also help learners distinguish between phonemic and quality phonemic while listening and differentiating, as well as correct phonemic errors, thereby increasing their language learning capacity. In order to study the application of nonlinear network identification technology in English learning, this paper evaluates the English pronunciation quality through the deep learning algorithm of deep learning combined with the related contents of neural network data model, and the experimental results of speech recognition structure are analyzed and discussed in detail. The concordance between machine and manual intonation evaluation is 80%, the concordance rate of adjacent intonation evaluation is 98.33%, and the Pearson correlation coefficient is 0.627 that shows the technique is reliable. The method of English pronunciation and speech identification model is sensible and dependable, which can give beginners a punctual, exact and impartial judgment and response guidance, assist learners to get on the differences between their phonemic and standard phonemic, and correct phonemic mistakes, in order to enhance the ability of oral English learning.

## 1. Introduction

Machine-learning technology controls numerous elements of modern life, from Internet searches to social media, content filtering to e-commerce web suggestions, and it is progressively present in consumer items such as cameras and smart phones. Machine-learning algorithms are used to recognize objects in photos, convert voice into text, match news articles, messages, or products with interests for users, and choose appropriate search outcomes [1, 2]. With the globalization and the improvement of China's internationalization level, the desire of the Chinese people for English learning is increasing day by day. However, due to the significant difference between Chinese and English pronunciation features, the domestic English learning environment remains untapped.

The article "Nonlinear Network Speech Recognition Structure in a Deep Learning Algorithm" was published in 2022. Journal: Comput Intell Neurosci.

There is a dearth of English teachers, and traditional classroom instruction cannot meet the needs of English learners owing to time and place constraints, among other things. All kinds of reasons have caused English teaching and learning become a major problem that puzzles the Chinese people, and English learning has also become one of the research hotspots in the discipline of education. As computer science and telecommunications develop the progress of language teaching and learning methods, the computer-aided language learning (CALL) technology makes it possible to solve this problem [3]. Computer-assisted language learning (CALL) is a method of teaching and learning in which the content to be learnt is presented, reinforced, and assessed using computer and computer-based resources such as the Internet. It generally has a significant interactive component. It also involves the search for an investigation of language teaching and learning applications. Except for self-study software, CALL is intended to augment rather than replace face-to-face language training [4, 5]. This technology will convert the continuing language educating method and learning environment and enable learners to learn independently at any moment and at any place, which can not only provide learners exact, target, and punctual phonemic estimation and response counselling. It can also help learners to get to the difference in the middle phonemic and quality phonemics along with reprise listening and differentiating and accurate their phonemic mistakes, thus improving the ability of language learning [6].

With the rapid growth in globalization, the people of China are learning the English language very rapidly. However, there is a shortage of English teachers in the region which causes a problem and creates considerable barriers. To overcome these issues, a deep learning-based algorithm is proposed which will not only check the English pronunciation but can also assist learners in distinguishing between their phonemic and quality phonemics when listening and differentiating, as well as correcting their phonemic errors, hence boosting their language learning capacity.

## 2. Literature Review

The construction of a neural network knowledge transmission processing system for deep learning is based on the application mode of the traditional neuron simulation information processing system, which is further improved and developed. The consistent system design of English phonemic learning and educating will gradually present a layered development model in the implementation of English phonemic aspects and voice knowledge identification and authentication. On the basis of combining with the neural construction model of deep learning, the professional teachers of English major in the discipline of education and research, it is clearly pointed out that the dominant style of this network construction is the solitary belonging education type [7]. Deep learning will have a lot of favorable outcome in near upcoming because it requires very little manual engineering and can easily take dominance of increases in computing and data availability. Neural network-based learning methods and architecture are being developed, which will only accelerate this process [8, 9]. It is important to integrate the learning method for speech recognition systems into it to obtain a knowledge-based interaction in those applications. The intelligent process can have feature extraction for further developed recognition process. The researcher acknowledges in integrating phonetic word units and pattern units with the acoustic process to achieve the best results in the speech recognition process [10]. English is one of the widely used languages, with the shrinking of the global village, the smart home, the in-vehicle voice system, and voice recognition software with English as the recognition language has gradually entered people's field of vision, and has obtained the majority of users' love by practical accuracy. Moreover, deep learning technology in many tasks with its hierarchical feature learning ability and data modeling capabilities has achieved more than the performance of shallow learning technology [11]. Based on the autonomous learning and unsupervised, a distinct number of system extent designs should stay in the manufacturing technique of up to seven layers to ensure the multilayer network building of deep learning, the system advantages reflected in the practical application process. To assure the multilevel network building of deep learning, the system advantages reflected in the practical application process, a distinct number of system extent architectures should remain in the manufacturing technique of up to seven layers. On the reasoning of comprehensively combining the data results of low-level knowledge, developing the transcoded English speech identification data belongs to a more ideal attribute classification. When required, the staff can also enhance the implementation ability of the great learning neural network architecture system by applying the analytical technique of distributed information layout. After long-term attempts and explorations by professionals in the same field, on the essential content of the new deep learning neural network construction mode, systematic and theoretical research conclusions are drawn. Professional researchers believe that implementing neural network knowledge processing mode from the perspective of deep learning essentially means combining the approach of multilevel mechanical learning tools with intensive exercises in English speech recognition and modulation training to help specify service teaching objects. By amending the management intensity of pronunciation training, the students' cognitive ability of the pronunciation learning effect is better demonstrated on the reasoning of understanding the analytic rules of phonemic learning. In the whole educational process of deep pronunciation, quality and recognition system building and implementation, the construction of deep model is the main way to describe the system functioning. Helping students to train and learn rational pronunciation depending on the characteristics of English pronunciation is the main teaching implementation aim of the deep learning framework model.

The article "Nonlinear Network Speech Recognition Structure in a Deep Learning Algorithm" was published in 2022. Journal: Comput Intell Neurosci.

In the aspect of pronunciation quality evaluation in China, the Institute of Automation, the Chinese Academy of Social Sciences, the University of Science and automation of China, Tsinghua University, and Microsoft Research Asia and Anhui Iflytek Co., Ltd conducted relevant research and have achieved corresponding results. The prosody factors are added to the original monophonic and triphone models, and the prosody model method is constructed, thus improving the pronunciation quality evaluation performance. Zhao et al. solved the confusion between probability space and target pronunciation acoustic model by studying the posterior probability of phoneme-related frame regular logarithm and its transformation, which made the pronunciation quality evaluation performance significantly improve [12]. Previous machine learning algorithms were limited in their ability to analyze natural data in their raw form. Designing a characteristic extractor that transforms raw data (such as image pixel values) into an appropriate internal state or feature vector from which the learning subsystem, often a classifier, could detect information has been collected in the insight required careful design and substantial domain expertise for centuries [13, 14]. Zoughi and Homayounpour put forward a new algorithm which introduces the GMM-UBM model into phoneme pronunciation quality evaluation and constructs a phoneme-independent feature distribution model [15]. The scoring effect is greater than the like algorithms, and it is near to skilled scoring relevance. Wang et al. put forward a new computing strategy, applying linguistic rules in the logarithmic posterior probability algorithm, and the correlation between machine scoring and manual scoring reached 0.795. Compared with the original algorithm, it is improved by 9% [16]. The evolution of speech-based machine learning has led to the development of a deep neural web, which is comparable to a neural network. The deep belief network (DBN) is one of the deep neural network techniques. Many researchers have devoted a significant amount of effort researching the usefulness of deep networks in modeling complex statistical events. According to the deep belief network theorem, the preferred learning approach in DBNs is a deep architecture network developed in RBM [17, 18]. Mazda et al. proposed a comprehensive evaluation algorithm of pronunciation quality reasoning on MFCC and LSP framework and the target scoring algorithm reasoning on elliptical model, which greatly enhanced the fairness and rationality of pronunciation attribute evaluation [19]. Higher computational power, more training data, and better software development have all given to the rapid victories of deep neural networks, in inclusion of improved learning methods. The initial breakthrough in acoustic modeling was due to the use of a generative texture before method for sensibly initializing the weights before running the discriminative back-propagation learning method, but subsequent research has revealed that generative pretraining is dispensable when there is a large amount of annotated training data [20, 21]. Yu et al. put forward a new pronunciation quality evaluation algorithm-PASS, and successfully applied to the CALL system for English learners the interactive language learning system in Tsinghua University. The sentence-level correlation between PASS and expert scoring is 0.66, which is superior to other scoring algorithms [22]. By differentiating the intonation speed, stress, rhythm, and intonation between the sentence to be evaluated and the standard sentence of corpus Hachuel made a comprehensive evaluation of pronunciation quality and achieved good results [23]. These research results provide strong support for the research and application of CALL. To sum up, the concept of deep learning is very popular at present. It provides high accuracy and high-speed calculation for speech recognition and creates new opportunities for intelligent speech interaction, so it has been widely recognized by academia and industry [24, 25].

The article "Nonlinear Network Speech Recognition Structure in a Deep Learning Algorithm" was published in 2022. Journal: Comput Intell Neurosci.

Conclusively, convolution neural networks are widely used in computer vision and have had a lot of success. They first showed promise for acoustic modeling but were later abandoned due to the fact that the convolution was done over time rather than frequency.

## 3. Research Methods

In this research, the neural network method of deep studying is adopted, and the Spoken Arabic Digit data fix in UCI machine learning library includes 8800 Arabic numerals (88 people pronounce 10 Arabic numerals and each numeral repeats 10 times), with 6600 pronunciations of the first 66 people as the training fix and 2200 phonemic of the last 22 people as the test set. The experimental software is Matlab R2013a.

### 3.1. Data Preprocessing

For neural networks, most of them have time regularity problems. Because the structure of the neural network classifier is fixed, and the length of the input speech signal is irregular, that is, the extracted speech attribute parameters have unequal dimensions, so we must transform the irregular length speech characteristic parameters into characteristic vectors with the similar length. In this paper, a piecewise mean method is used to preprocess the speech feature parameters of Spoken Arabic Digit data set, such as dimension reduction and regularization. First, the feature parameters of the speech signal are segmented on average, which can be expressed as *JKS*, where *K* is the order of feature parameters, *J* is the frame number of segmented feature parameters, and *T* is the original speech frame number. Formula (1) for dividing the characteristic parameters into *n* segments on average is as follows:

(1) $$\begin{array}{c} M\left(i\right)=S\left(K,J\right),J=\left[\frac{T}{N}\left(i=1\right)+1\right],\ldots ,\left[\frac{T}{N}i\right]. \end{array}$$

*M*(*i*) is the speech characteristic framework of the segment after segmentation. In this paper, the value of *n* is 4, which can be taken according to the actual needs in practical application, but its value is restricted by the feature dimension of the speech signal. After the characteristic parameters are averagely divided into *N* segments, *M*(*i*) is averagely divided into *M* segments. In this paper, the value of *M* is 3, which is constrained by the dimension of speech feature together with *N*. and then average frame parameters of each subsegment to get the mean vectors *M*_k1_, *M*_k2_,… *i* of each subsegment. After obtaining the mean vector of each subsegment, the mean values of each subsegment are combined into a matrix, that is, the matrix TKS with the size of NMK is obtained, and TKS, TKS are the output values of characteristic parameters after dimension reduction and regularization. The segmentation, mean reduction, and regularization of speech feature parameters are shown in Figure 1.

The article "Nonlinear Network Speech Recognition Structure in a Deep Learning Algorithm" was published in 2022. Journal: Comput Intell Neurosci.

Because the input speech can be irregular and may have unequal dimensions; Figure 1 clearly depicts the block diagram for improving speech improvement and to convert into characteristic vectors with the similar length. It will also help with dimension reduction and regularization.

The total number of speech characteristic parameters at each stage in Figure 1 is shown in Table 1.

The piecewise mean dimension reduction regularization algorithm can reduce the dimension of the KT-sized characteristic parameter matrix to an NMK-sized parameter matrix. According to the formula, NMK, the piecewise mean dimensionality reduction regularization algorithm, successfully removes the influence of speech frame number *t* on the data size after dimensionality reduction regularization, and the parameter matrix size after dimensionality reduction regularization is only related to the characteristic parameter order *k*, the subsection size *n,* and the subsection size *m*. It makes every speech with different lengths be regularized into a matrix with the same size, which greatly facilitates the realization of speech recognition algorithm and greatly improves the performance of speech recognition algorithm.

In this observation, every speech signal is normalized to 16 frames, that is, the data amount of every presentation signal is 13∗16 = 208. Furthermore, the normalized Spoken Arabic Digit data set after dimensionality reduction is [0,1], which is beneficial to reduce the influence of feature differences caused by different speakers and channels. In addition, the deep neural network uses small batch data processing to reconstruct the error adjustment weights, make the network more stable, and run more efficiently. However, the data set has a certain order, so it is necessary to randomly scramble the data set before batch processing to enhance the performance of the model.

## 4. Research Results

### 4.1. Result Analysis

This technology will revolutionize the current language teaching technique and learning environment, allowing students to learn independently at any time and in any location. It will not only give learners with exact, targeted, and timely phonemic estimation and response guidance but it will also let them to study autonomously at any time and in any location. The proposed deep learning model has been compared with other various models for the recognition rate. The detailed results have been shown in the table form. Meng et al. [26] proposed a new tree distribution approximation model based on the graph tree structure (TDA-GTS) for the same Spoken Arabic Digit data fixed in UCI artificial learning library, and compared it with TDA-MWST, DHMM, and CDHMM. Huang Wen Tao proposed a *K*-means clustering method found on selective weights and thresholds (KASWT), and compared with BP_Adaboost algorithm, the recognition effect was improved. Here, the model in this paper is compared with the above models, and the contrast results of identification rate are shown in Table 2.

The article "Nonlinear Network Speech Recognition Structure in a Deep Learning Algorithm" was published in 2022. Journal: Comput Intell Neurosci.

It is noticed from Table 2 that the recognition rate of DBN model constructed in this paper is 96.64%, which is better than the above model. Therefore, the representation recognition model is construct based on DBN established in this paper, is suitable and effective, and can further be used in the estimation of pronunciation quality.

### 4.2. English Speech Recognition Evaluation Process under Deep Learning

According to the perspective of deep learning, the practice starting point and cognitive angle of English pronunciation quality evaluation are different. The existing types of pronunciation quality evaluation can be further divided into subjective evaluation and objective evaluation. Subjective evaluation in English pronunciation quality refers to the evaluation activities carried out by language expression experts according to their accumulated professional pronunciation. Under normal circumstances, the evaluation of pronunciation quality in this form should strictly follow the cognitive impression of the evaluators themselves. By testing the sound quality of pronunciation courseware, the examiners compare and evaluate the English pronunciation of the examinees according to their accumulated pronunciation cognition. In the process of comprehensive evaluation, different conclusions are drawn, and different numbers of comprehensive evaluation scores are given.

The factual test is a process of assessing the standard of English pronunciation that is not based on interpretive evaluation activities. There is a significant difference between quantitative and qualitative evaluation. The application of the ranking tools necessitates the use of various types of mechanical review instrumentation. The metrics and establishing of different assessment scores are governed under the scanning feature of artificial intelligence information system operation in the practice of instantaneous and impartial phonemic quality assessment. In comparison to the frequency of judgment mistakes in incentive judgment, the use of an external validation mode could much more deeply portray the impartiality of phonemic internal audits. The procured standard evaluation conclusion can also better meet the expert of prime admission organizations and investigation planners.

The article "Nonlinear Network Speech Recognition Structure in a Deep Learning Algorithm" was published in 2022. Journal: Comput Intell Neurosci.

According to the method described in this paper, the scores of pitch, speech speed, rhythm, and intonation of 24 students with 10 sentences and 240 sentences can be obtained, which are further compared with manual evaluation. The experimental outcomes are shown in Tables 3 and 4.

In the pitch evaluation, there seem to be 207 specimens who have the same grade as employee evaluations, 32 accessions that vary by one grade, one sample that varies by different grades, and thus no samples that differ by three levels. It exemplifies that the exactness of equipment and routine tonality review is 86.25 percent, the adjacent prediction accuracy is 99.58 percent, and the Pearson correlation is 0.8, suggesting that the intonation review proposed method is accurate. In the words of speaker analysis, there are 197 samples which are the same level as employee evaluations, 43 specimens that differ through one level, and no specimen that differs by two or three levels. The constant rate of device and routine speed analysis is 87 percent, the adjoining constant rate has increased as 100 percent, and the Pearson's correlation coefficient is 0.493, suggesting that the speed analysis method employed in this study is convincing. There are 204 specimens with the same level of device and manual groove analysis, 33 samples with one gradient, only three specimens with two stages variation, and no specimens with three parameters differences; it reveals that the synchronization rate between the device and instructions groove analysis is 85 percent, the adjoined statistical quirk rate is expected to rise as 98.75 percent, and Pearson's correlation coefficient is 0.543, denoting that the ray. There are 192 samples of the same level of device analysis and manual analysis, 44 specimens by one gradient, only 4 specimens with two stages distinction, but no specimens with three parameters distinction in inflection analysis; it reveals that the constant rate of device and manual inflection analysis is 80 percent, the adjacent constant rate has increased as 98.33 percent, and the coefficient of correlation is 0.627, implying that its tonal assessor is accurate. To conclude, the performance measures shown in this paper for sound, speech frequency, rhymes, and tonality are credible that can be used to build a Listening and speaking product analysis approach.

The experimental results are shown in Figure 2. The number of tests with the similar level of machine evaluation and manual evaluation is consistent, and there is no difference in the number of samples with two or three levels; The overall coincidence rate of machine and manual evaluation is 90%, and the adjacent coincidence rate is as high as 100%, which shows that there is a powerful correlation between machine evaluation and manual evaluation.

The article "Nonlinear Network Speech Recognition Structure in a Deep Learning Algorithm" was published in 2022. Journal: Comput Intell Neurosci.

## 5. Conclusions

With the help of modern computer information processing technology, English pronunciation quality evaluation and deep learning of speech recognition have found the R&D core that can promote its rapid development. At present, the technical staff in the same field in China, based on the basic concept of pronunciation neural network recognition system, the system construction mode of deep learning neural network is developed. Technicians can objectively judge the framework effect of English pronunciation quality from the perspective of deep learning and deeply study the deep learning method to improve the speech recognition effect. The results shows that the device and manual inflection analysis constant rate is 80%, the adjacent constant rate has grown to 98.33%, and the coefficient of correlation is 0.627, meaning that the tonal assessor is accurate. To summarize, the sound, speech frequency, rhymes, and tonality performance metrics presented in this research are reliable and may be utilized to develop a listening and speaking product analysis strategy, continue to study the deep faith network, and enhance the accuracy and speed of speech identification. On this basis, we try to study more deep learning algorithms, such as depth automatic encoder and convolutional neural network, and compare the advantages and disadvantages of various algorithms to find out the better algorithms and models. It is sure that with the rapid development of hardware and processing technologies, neural networks will attract more attention and find more applications in the future.

## Figures and Tables

**Figure 1:** Schematic diagram of segmentation, mean dimension reduction, and regularization of speech characteristic parameters.

**Figure 2:** Overall evaluation differences between machine and labor.

**Table 1:** Number table of segmented mean dimension reduction and regular parameters of speech characteristic parameters.

Parameter condition	Stage					
	I	II	III	IV	V	VI
Matrix size	T∗K	(T/N)∗K	(T/(M∗N))∗K	([T/(M∗N)]∗[1/T/(M∗N)])∗K	M∗K	(M∗N)∗K
Number of parameters	T∗K	T∗K	T∗K	K∗M∗N	K∗M∗N	K∗M∗N

**Table 2:** Comparison of recognition rates under different models.

Indicators	
Model	Discrimination (%)
DHMM	90.79
CDHMM	94.09
TDA-MWST	93.16
TDA-GTS	93.09
BP-Adaboost	89.37
KASWT	92.68
This model	96.64

**Table 3:** Evaluation index experimental results-number of samples.

Indicators	Number of samples (pieces)			
	Consistent	The difference is one level	The difference is two levels	The difference is three levels
Accuracy in pitch	207	32	1	0
Speed	197	43	0	0
Rhythm	204	33	3	0
Intonation	192	44	4	0

The article "Nonlinear Network Speech Recognition Structure in a Deep Learning Algorithm" was published in 2022. Journal: Comput Intell Neurosci.

**Table 4:** Evaluation index experimental results-statistical indicators.

Indicators	Difference level		
	Consistency rate (%)	Adjacent coincidence rate (%)	Pearson
Accuracy in pitch	86.25	99.58	0.8
Speed	82.08	100	0.493
Rhythm	85.00	98.75	0.543
Intonation	80.00	98.33	0.627

## Data Availability

The data used are available from the corresponding author upon request.
